The article "Investigation on the Effect of Graded Emergency Nursing Group under the Assistance of Multidisciplinary First Aid Knowledge Internet-Based Approach on the First Aid of Acute Myocardial Infarction" was retracted in 2023. Reason: concerns about the peer review.

# Investigation on the Effect of Graded Emergency Nursing Group under the Assistance of Multidisciplinary First Aid Knowledge Internet-Based Approach on the First Aid of Acute Myocardial Infarction

**DOI:** 10.1155/2022/8469930

**Published:** 2022-01-18

**Authors:** Lili Song, Han Lu, Hong Ru, Xue Zhao

**Affiliations:** Department of Emergency, Beijing Hospital, National Center of Gerontology, Institute of Geriatric Medicine, Chinese Academy of Medical Sciences, No.1 Da HuaRoad, DongDan, Beijing 100730, China

## Abstract

**Objective:**

To analyze the effect of a graded emergency nursing group under the assistance of multidisciplinary first aid knowledge Internet-based approach on the first aid of acute myocardial infarction (AMI).

**Methods:**

The clinical data of 90 AMI patients treated in our hospital from March 2019 to March 2020 were selected for the retrospective analysis, and the patients were divided into the observation group and the routine group according to the first aid order, with 45 cases each. The patients in the routine group received the conventional first aid measures, and the graded emergency nursing group mode with the help of multidisciplinary first aid knowledge Internet-based approach was adopted for those in the observation group so as to compare the prognosis, nursing satisfaction scores, etc., between the two groups.

**Results:**

Compared with the routine group, patients in the observation group obtained significantly lower various fast reaction indicators and quality of life score (*P* < 0.001), higher nursing satisfaction score (*P* < 0.001), lower total complication rate (*P* < 0.05), higher successful rescue rate (*P* < 0.05), and lower AMI recurrence rate and PCI reuse rate (*P* < 0.05).

**Conclusion:**

Rescue measures by the graded emergency nursing group with the help of multidisciplinary first aid knowledge Internet-based approach are a reliable method for improving AMI patients, and such strategy greatly promotes patients' quality of life and reduces the PCI reuse rate. Further research will be conducive to establishing a better solution for AMI patients.

## 1. Introduction

Acute myocardial infarction (AMI), the myocardial ischemic necrosis resulting from the blockage of coronary arteries, is a common critical illness with the characteristics such as rapid disease progression, poor clinical prognosis, and high mortality [1, 2]. Early reperfusion is the key to rescuing patients, and studies have found that [3] the case fatality rate reaches 6% in those who received reperfusion with onset >6 h and decreases to 2% in those who received reperfusion with onset <1 h, indicating that prompt rescue is significant in reducing the mortality of AMI patients [4, 5]. Routine first aid processes are cumbersome and significantly delay the rescue time, so optimization is necessary [6, 7]. For patients with critical, urgent, and complex condition, instead of single department working alone, multiple departments must jointly carry out first aid by the way of consultation to exploit their advantages to the full, thereby taking effective first aid measures with the shortest time and improving the success rate of first aid to the greatest extent through close cooperation. With the help of the modern Internet assistance model, an emergency network consisting of the emergency center, clinic, community medical service, primary hospital, and ambulance is connected, thus helping rescue staff to drive out to the emergency scene precisely and quickly and greatly reducing the time from patients' onset to admission. The treatment effect has been proved in the first aid of severe craniocerebral trauma and chest pain [8]. In addition, investigations found that triage and first aid for patients with different degrees of critical diseases can maximize the first aid efficiency of nurses at different grades and that the implementation of graded first aid nursing in the rescue process can effectively shorten the rescue time, which has been confirmed in the rescue of patients with abdominal trauma accompanied by hemorrhagic shock [9]. At present, there are fewer reports about the graded emergency nursing group with the help of multidisciplinary first aid knowledge Internet-based approach in the first aid of AMI, and the following study was carried out on the basis of the background.

The article "Investigation on the Effect of Graded Emergency Nursing Group under the Assistance of Multidisciplinary First Aid Knowledge Internet-Based Approach on the First Aid of Acute Myocardial Infarction" was retracted in 2023. Reason: concerns about the peer review.

## 2. Materials and Methods

### 2.1. General Data

The clinical data of 90 AMI patients treated in our hospital from March 2019 to March 2020 were selected for the retrospective analysis, and the patients were divided into the observation group and the routine group according to the first aid order, with 45 cases each. The study met the World Medical Association Declaration of Helsinki (2013) [10].

### 2.2. Inclusion and Exclusion Criteria

Inclusion criteria were defined as follows: (1) the patients who were diagnosed with AMI by coronary angiography, with clinical manifestations including severe angina, dizziness, dyspnea, and vomiting, and received first aid treatment within 12 h upon onset; (2) the patients who presented classic changes of myocardial enzymes of AMI (abnormal troponin, creatine kinase isoenzyme, and myoglobin levels); and (3) the patients who had good mental status and could cooperate with the treatment.

Exclusion criteria were defined as follows: (1) the patients who had chronic obstructive pulmonary disease (COPD) and severe mental diseases or were complicated with severe dysfunction in the liver, kidney, and other organs; (2) the patients who had a history of chronic heart disease or heart surgery; and (3) the patients who were complicated with cardiac insufficiency or language expressing difficulty.

The article "Investigation on the Effect of Graded Emergency Nursing Group under the Assistance of Multidisciplinary First Aid Knowledge Internet-Based Approach on the First Aid of Acute Myocardial Infarction" was retracted in 2023. Reason: concerns about the peer review.

### 2.3. First Aid Measures

The patients in the routine group accepted the traditional first aid mode. After admission, the blood test was performed on patients in time, two or three effective vein passages were opened as early as possible, patients were guided to rest in bed, and continuous electrocardiographic monitoring was conducted to closely monitor changes in various vital signs and carefully observe patients' condition. After the patients were diagnosed, the nurses prepared the patients for surgery and sent them to the catheterization room [11, 12].

The graded emergency nursing group mode under the assistance of multidisciplinary first aid knowledge Internet-based approach was conducted on patients in the observation group with the following specific steps. (1) An emergency nursing group consisting of 1 head nurse, 2 senior nurses, 5 nurses, and 2 specialist physicians was set up with the head nurse as the group leader. The emergency nurses were graded, to be specific, those with at least 5 years of working experience and obtained the professional title of above senior nurse were primary nurses; those with at least 3 years of working experience and obtained the professional title of nurse or senior nurse were secondary nurses; and the nurses, practice nurses, or senior nurses engaged in advanced studies with less than 3 years of working experience were tertiary nurses. (2) A regional Internet collaborative treatment mode for AMI was established. With the help of the “BianQueFeiJiu” remote emergency system and the AMI WeChat group, physicians of the community clinic, emergency clinic, and our hospital could quickly send patients' ECGs to our AMI emergency center and perform online communication, realizing disease recognition and consultation in a timely manner. The “BianQueFeiJiu” information-based system was equipped in ambulance that enabled the use of wireless 12-lead ECG monitor, oximetry, glucometer, etc., to monitor patients' various vital signs and transmit these data and site rescue video to our AMI emergency center via 4G satellite channel in real time so that the experts of the emergency center could carry out consultation on patients' sudden condition in advance based on the data and video and timely provide relatively reasonable guidance on first aid, and patients admitted to the primary-level medical unit of remote area or on the way to the hospital could receive treatment from our hospital in advance. (3) Weekly multidepartment assistance training was carried out to members of the group with the following contents. First, the group leader clarified the training key points and objectives; second, the director of the department of cardiology explained the clinical manifestations, diagnosis, and first aid key points of AMI with specific cases in detail, focusing on helping the emergency nurses to master relevant AMI knowledge; third, based on the selected cases, the director of emergency department explained the diagnosis, first aid, relevant examinations, escort, preoperative preparation, etc., in the first aid of AMI, nursing key points, and relevant precautions of various links and handing over to the catheterization room in detail; and finally, the head nurse of cardiac care unit explained the relevant nursing operation of patients in the unit by referring to classic cases and demonstrating on-site operation. Members of the group raised questions about the problems that occurred during first aid based on the explanation of each department. According to the training and possible problems, the group leader did in-depth organization and analysis, discussed with experts of other departments, optimized and improved various links of first aid in combination with the opinions of other group members, and established a new standardized first aid process.

The article "Investigation on the Effect of Graded Emergency Nursing Group under the Assistance of Multidisciplinary First Aid Knowledge Internet-Based Approach on the First Aid of Acute Myocardial Infarction" was retracted in 2023. Reason: concerns about the peer review.

### 2.4. Observation Indexes

Fast response indicators: the time from onset to admission, admission to the completion of first myocardial enzyme examination, first medical contact to vascular opening, and onset to calling 120 patients in the two groups was recorded.

After the patients' condition was stable, the satisfaction of the clinical care of AMI patients in our emergency center was investigated with the questionnaire made by our hospital, which contained 4 items, namely, reception operation, basic nursing, service attitude, and service quality. On a scale of 0–100 points, higher scores indicated higher patient satisfaction on clinical emergency care.

The quality of life of patients in the two groups was assessed by the myocardial infarction dimensional assessment scale (MIDAS) [13], which included 7 dimensions (emotional reaction, security, diet, physical activity, dependency, worry about medication, and adverse drug reactions) and 35 items. Each item was rated by the 5-grade scoring method (0–4 points), and higher scores indicated the worse quality of life.

Prognosis: the successful rescue rate, AMI recurrence rate, and PCI reuse rate of the two groups were observed and recorded.

The occurrence of complications of the two groups was recorded, which included arrhythmia, cardiogenic shock, chest pain, and hypotension.

The article "Investigation on the Effect of Graded Emergency Nursing Group under the Assistance of Multidisciplinary First Aid Knowledge Internet-Based Approach on the First Aid of Acute Myocardial Infarction" was retracted in 2023. Reason: concerns about the peer review.

### 2.5. Statistical Methods

In this study, the data were processed by the professional statistical software SPSS23.0, the picture drawing software was GraphPad Prism 7 (GraphPad Software, San Diego, USA), the enumeration data were examined by the *X*^2^ test and expressed by (*n*(%)), the measurement data were examined by the *t* test and expressed by mean ± SD, and differences were considered statistically significant at *P* < 0.05.

## 3. Results

### 3.1. Comparison of Clinical Data

No statistical differences in general data including the mean age, blood pressure value, infarction site, and place of residence between the two groups were observed (*P* > 0.05) (see Table 1).

### 3.2. Comparison of Rapid Response Indicators

Various fast response indicators were significantly lower in the observation group than in the routine group (*P* < 0.001) (see Table 2).

### 3.3. Comparison of Nursing Satisfaction Scores

The nursing satisfaction score was significantly higher in the observation group than in the routine group (*P* < 0.001) (see Figure 1).

### 3.4. Comparison of Quality of Life Scores

The quality of life score was significantly lower in the observation group than in the routine group (*P* < 0.001) (see Figure 2).

### 3.5. Comparison of Prognosis

Compared with the routine group, the observation group obtained significantly higher successful rescue rate (*P* < 0.05) and significantly lower AMI recurrence rate and PCI reuse rate (*P* < 0.05) (see Table 3).

### 3.6. Comparison of Complication Rates

The total complication rate was significantly lower in the observation group than in the routine group (*P* < 0.05) (see Table 4).

## 4. Discussion

AMI is a symptom of myocardial necrosis due to acute, sustained ischemia and hypoxia in coronary arteries, which is often complicated by arrhythmias, heart failure, and other complications, seriously threatening the life health of patients [14]. Several studies have confirmed that, for AMI patients, the implementation of timely and effective care is a key to reducing mortality and improving the quality of survival [15–17]. Conventional first aid models are often less normative and methodical and tend to make mistakes in the actual on-site rescue process with low efficiency, resulting in poor patient outcomes. With the rapid development of Internet technology in recent years, the “Internet + smart first aid” mode has been established in hospitals, which integrates modern Internet communication technology into clinical first aid, breaks through the spatiotemporal limitations of traditional prehospital rescue medical activity, better achieves prehospital and in-hospital seamless docking, and greatly eliminates the rescue blind area [18]. AMI patients have an urgent and complex condition, which requires multiple departments to carry out a common rescue treatment by the way of consultation, which has achieved the expected effect in the first aid of AMI [19, 20]. The reasons are as follows: (1) In the rescue and treatment modes, the diagnosis and treatment of various departments are conducted independently, so the departments cannot timely communicate on the information of clinical diagnosis and understand the patients' condition, often leading to missing the optimal treatment timing and extending the time of rescue treatment. (2) The multidepartment model of first aid has multiple roles from multiple departments and is able to ensure that, during the process of rescuing patients, the operation of the organization is not affected by external factors, thereby greatly enhancing the rescue effect [21]. Graded first aid triages patients separately from different grades of critical care such that nurses with different grades exert the greatest first aid efficiency, which has been proved in the first aid of patients with critical cardiovascular disease in the emergency department [22]. By reviewing relevant information and combining it with clinical first aid emergency, the study achieved better rescue outcomes by implementing graded acute care group rescue measures assisted by a multidisciplinary emergency knowledge Internet-based approach for AMI patients.

The article "Investigation on the Effect of Graded Emergency Nursing Group under the Assistance of Multidisciplinary First Aid Knowledge Internet-Based Approach on the First Aid of Acute Myocardial Infarction" was retracted in 2023. Reason: concerns about the peer review.

The comparison of various indices of rapid response between the two groups revealed that, compared with the routine group, the indices such as time from onset to admission and from first medical contact to vascular opening were significantly lower in the observation group, and the reason was that such care model well solved the problems such as delays in hospital care. This care model can connect emergency centers, clinics, medical service stations, ambulance, etc., into a single emergency network, which maximally extends advanced rescue technology to the front line and better achieves synergistic first aid of AMI, thus effectively avoiding under- or overtreatment, which has been confirmed in the rescue of patients with acute cerebral hemorrhage [23]. The study results showed that the nursing satisfaction score was significantly higher in the observation group than in the routine group, indicating that the graded emergency nursing group with the assistance of multidisciplinary emergency knowledge Internet-based approach could greatly improve patients' nursing satisfaction, and the reason was that group members performed their own tasks during the process of rescue, implemented comprehensive care to patients based on the first aid knowledge of AMI they had mastered, and obtained the recognition from patients and their family members because of their solid expertise and operational skills and high-efficient group care, thus enhancing the satisfaction [24, 25]. Shortcomings of the study are as follows: due to the limited study conditions, the study had a smaller sample size and single case source, and the effect of factors such as disease classification on study results was not considered, so the specific rescue plan should be constantly summarized and improved in future clinical practice.

The article "Investigation on the Effect of Graded Emergency Nursing Group under the Assistance of Multidisciplinary First Aid Knowledge Internet-Based Approach on the First Aid of Acute Myocardial Infarction" was retracted in 2023. Reason: concerns about the peer review.

## Figures and Tables

**Figure 1:** Comparison of nursing satisfaction scores between the two groups (mean ± SD). Note: the horizontal axis indicates the observation group and the routine group, and the vertical axis indicates the nursing satisfaction score in points; the nursing satisfaction scores of the observation group and the routine group were (83.16 ± 4.73) and (83.16 ± 4.73); ^*∗*^ indicates a significant difference in the nursing satisfaction scores between the two groups (*t* = 6.999; *P* < 0.001).

**Figure 2:** Comparison of the quality of life scores between the two groups (mean ± SD). Note: the horizontal axis indicates the observation group and the routine group, and the vertical axis indicates the quality of life score in points; the mean quality of life scores of the observation group and the routine group were (38.44 ± 6.28) and (42.44 ± 6.69); ^*∗*^ indicates a significant difference in the mean quality of life scores between the two groups (*t* = 2.924; *P* < 0.05).

**Table 1:** Comparison of clinical data.

Item	Observation group	Routine group	*X* ^2^/*t*	*P*
Gender			0.044	0.833
Male/female	23/22	22/23		
Body mass index (kg/m^2^)	22.16 ± 5.38	22.21 ± 5.27	0.045	0.965
Mean age (mean ± SD, years)	61.26 ± 3.26	61.32 ± 3.31	0.087	0.931
Mean course of disease (mean ± SD, h)	3.02 ± 0.24	3.04 ± 0.31	0.342	0.733
Blood pressure value (mmHg)				
Systolic blood pressure	136.22 ± 8.25	136.31 ± 8.19	0.052	0.959
Diastolic blood pressure	82.15 ± 6.28	82.24 ± 6.24	0.068	0.946
Renal function indicator				
Urine nitrogen (mmol/L)	6.23 ± 0.73	6.27 ± 0.65	0.275	0.784
Creatinine (*μ*mol/L)	82.16 ± 11.23	82.21 ± 11.18	0.021	0.983
Infarction site				
Inferior wall	14 (31.11%)	15 (33.33%)	0.051	0.822
Anterior wall	12 (26.67%)	14 (31.11%)	0.216	0.642
High lateral wall	19 (42.22%)	16 (35.56%)	0.421	0.517
Blood lipid (mmol/L)				
Triacylglycerol	1.46 ± 0.25	1.42 ± 0.28	0.715	0.477
Cholesterol	4.62 ± 0.41	4.71 ± 0.52	0.912	0.364
Educational degree				
College	3 (6.67%)	5 (11.11%)	0.549	0.459
High school	12 (26.67%)	13 (28.89%)	0.055	0.814
Primary school	30 (66.67%)	27 (60.00%)	0.431	0.512
Place of residence			0.180	0.671
Urban area	19 (42.22%)	21 (46.67%)		
Rural area	26 (57.78%)	24 (53.33%)		

The article "Investigation on the Effect of Graded Emergency Nursing Group under the Assistance of Multidisciplinary First Aid Knowledge Internet-Based Approach on the First Aid of Acute Myocardial Infarction" was retracted in 2023. Reason: concerns about the peer review.

**Table 2:** Comparison of rapid response indicators (mean ± SD, min).

Group	*n*	Time from onset to admission	Time from admission to the completion of first myocardial enzyme examination	Time from first medical contact to vascular opening	Time from onset to calling 120
Observation	45	54.27 ± 14.26	13.27 ± 3.26	89.46 ± 10.17	20.23 ± 5.26
Routine	45	66.23 ± 11.34	24.27 ± 3.31	117.23 ± 9.27	36.17 ± 5.18
*t*		4.404	15.883	13.537	14.484
*P*		<0.001	<0.001	<0.001	<0.001

**Table 3:** Comparison of prognosis between the two groups (*n*(%)).

Group	*n*	Successful rescue rate	AMI recurrence rate	PCI reuse rate
Observation	45	100 (45/45)	2.22 (1/45)	0 (0.00)
Routine	45	91.11 (41/45)	13.33 (6/45)	8.89 (4/45)
*X* ^2^		4.186	3.873	4.186
*P*		<0.05	<0.05	<0.05

**Table 4:** Comparison of complication rates between the two groups (*n*(%)).

Group	*n*	Arrhythmia	Cardiogenic shock	Chest pain	Hypotension	Total incidence rate
Observation	45	0 (0.00)	1 (2.22)	0 (0.00)	1 (2.22)	4.44% (2/45)
Routine	45	1 (2.22)	2 (4.44)	2 (4.44)	3 (6.67)	17.78% (8/45)
*t*						4.050
*P*						<0.05

## Data Availability

The data used to support the findings of this study are available on reasonable request from the corresponding author.
